RETRACTED

# A Neighborhood and Machine Learning-Enabled Information Fusion Approach for the WSNs and Internet of Medical Things

**DOI:** 10.1155/2022/5112375

**Published:** 2022-04-11

**Authors:** Zard Ali Khan, Sheneela Naz, Rahim khan, Jason Teo, Abdullah Ghani, Mohammed Amin Almaiah

**Affiliations:** ^1^Department of Computer Science, Comsats University, Islamabad, 45550, Pakistan; ^2^Faculty of Computing and Informatics, University of Malaysia Sabah, Malaysia; ^3^Department of Computer Science, Abdul Wali Khan University Mardan, Pakistan; ^4^Department of Computer Networks and Communications, College of Computer Sciences and Information Technology, King Faisal University, Al-Ahsa, Saudi Arabia

## Abstract

Data redundancy or fusion is one of the common issues associated with the resource-constrained networks such as Wireless Sensor Networks (WSNs) and Internet of Things (IoTs). To resolve this issue, numerous data aggregation or fusion schemes have been presented in the literature. Generally, it is used to decrease the size of the collected data and, thus, improve the performance of the underlined IoTs in terms of congestion control, data accuracy, and lifetime. However, these approaches do not consider neighborhood information of the devices (cluster head in this case) in the data refinement phase. In this paper, a smart and intelligent neighborhood-enabled data aggregation scheme is presented where every device (cluster head) is bounded to refine the collected data before sending it to the concerned server module. For this purpose, the proposed data aggregation scheme is divided into two phases: (i) identification of neighboring nodes, which is based on the MAC address and location, and (ii) data aggregation using *k*-mean clustering algorithm and Support Vector Machine (SVM). Furthermore, every CH is smart enough to compare data sets of neighboring nodes only; that is, data of nonneighbor is not compared at all. These algorithms were implemented in Network Simulator 2 (NS-2) and were evaluated in terms of various performance metrics, such as the ratio of data redundancy, lifetime, and energy efficiency. Simulation results have verified that the proposed scheme performance is better than the existing approaches.

## 1. Introduction

Internet of Things (IoT) consist of numerous sensor nodes, devices, and server(s), which are either deployed randomly or in deterministic fashion to probe the physical phenomena after a defined time interval [1]. However, due to their dense deployments, these networks often generate a huge volume of data, mostly redundant or duplicate, which is needed to be refined before the transmission activity is initiated either by a node or cluster head (CH) or server module. As a result, the ratio of the transmitted packets is increased, which is directly proportional to the lifetime of operational IoT networks. Data aggregation is one of the common approaches that is used to minimize the ratio of redundancy in data captured by sensor nodes residing in closed proximity [2, 3]. Furthermore, the transmission of these redundant data set without proper refinement leads to numerous challenges, that is, wastage of resources such as bandwidth, on-board battery, and congestion throughout the IoT networks [4]. Machine learning-based approaches are assumed among the promising techniques, which are utilized to address these issues preferably with the available resources and infrastructure.

RETRACTED

Generally, in Internet of things and resource-limited networks, communication activity is assumed as more energy starving than processing. Therefore, data captured by various sensor nodes should be refined, that is, the minimum possible ratio of the duplicate data or packets, before transmitting it to the intended destination module (i.e., base station or sink in this case). The data refinement process is carried out by an ordinary node (if WSNs are homogeneous) or CH or both if the underlined WSN is heterogeneous [5]. In both cases, the ultimate goal is to refine raw data captured by sensor nodes, which are called data aggregation or fusion. Thus, the size of the captured data set is reduced with a minimum possible ratio of information loss. Additionally, the number of packets needed to be transmitted by various source nodes is minimized by avoiding duplicate transmissions and, thus, enhances the overall lifespan of both individual node and the entire WSNs [6, 7]. In the literature, various data aggregation and fusion mechanisms are presented to address to aforementioned issue; however, the majority of these approaches are focused on how to control the communication cost as it is assumed as the main consumer of the on-board battery in the WSNs infrastructures [8, 9]. Apart from it, these approaches rely on the duplicate-insensitive functions, which are directly proportional to the duplicate value elimination time [10]. Additionally, the majority of the existing approaches are not sensitive to the duplicate or redundant data values and outliers, which are generated due to malfunctioning of an ordinary node, in the operational WSNs. A periodic clustering approach was proposed where the main objective was to improve transmission efficiency and eliminate data redundancy. This approach is based on two tiers: one is to eliminate redundancy in every period from sensing data if member nodes and the other is for one-way ANOVA model using the *k*-mean algorithm with three statistical tests to eliminate data redundancy from the participant that make redundant data sets [11]. These approaches are designed according to the resource-constrained nature of the sensor nodes and CH as a slightly higher computation and space overheads are energy starving. Therefore, data aggregation approaches designed for the WSNs should be energy and performance efficient [12]. In addition to it, the accuracy of the captured data is one of the common issues associated with the WSNs, which is usually due to the resource-constrained nature of member devices or sensor nodes [13]. Therefore, the design and development of the energy and performance efficient data aggregation approaches is still an open challenge both for the researcher and organizations. In this paper, energy- and performance-efficient data aggregation approach is presented to resolve the aforementioned issue, that is, duplication data value, with the available resources in the operational WSNs. For this purpose, a simplified distance measure is used to enable a dedicated CH to refine the collected data by eliminating duplicate data values. Furthermore, the proposed data aggregation scheme bound every CH to match data sets of a neighboring node only as it is quite likely that data captured by node reside in closed proximity are highly correlated than other nodes. For this purpose, the proposed data aggregation scheme is divided into two phases, which are given below.

1. Identification of neighboring nodes, which is totally based on their MAC address and location information.
2. Apply data aggregation using *k*-mean clustering and Support Vector Machine (SVM) algorithms.

RETRACTED

The proposed data aggregation scheme has restricted the concerned CH to refine data sets of those neighboring node that reside in vicinity (i.e., able to communicate directly with each other). The main contributions of this research work are as given below.

1. A MAC-enabled mechanism for the identification of neighboring nodes
2. A smart data aggregation approach for the resource's constraint networks, such as IoTs
3. Neighborhoods-enabled algorithm to avoid unnecessary matching of data values in the data aggregation process

The remaining of this paper is organized as follows. In Section 2, a brief but comprehensive literature review of data aggregation approaches is presented whereas Section 3 depicts a detailed explanation of the proposed scheme (i.e., neighborhood-enabled data) aggregation, which is based on cluster-based networking infrastructure. In Section 4, the proposed data aggregation algorithm with proper mathematical background is presented. In subsequent section, simulation results of proposed and existing approaches in terms of various performance metrics are presented. Finally, concluding remarks and future direction are provided.

RETRACTED

## 2. Related Work

Various approaches have been proposed in the literature for cluster-based data aggregation, such as *k*-mean clustering-based, Euclidean distance, cosine distance, one-way ANOVA model, Jaccard function, analysis of variance, and so on. The authors [14] presented the EK-means clustering approach for classification of data set to reduce the volume of sending data over the network. The approach is based on two steps: (i) elimination of data redundancy at sensor level using Euclidean distance measure and (ii) group similar data sets or values and, thus, minimizing the number of packets required to be sent using the EK-means approach. The author [15] has proposed a modified *k*-means approach to eliminate data redundancy and enhance the sensor network lifetime and forward minimum possible packets to the intended destination module that is the base station in this case. The authors [16] have proposed a *k*-mean clustering data aggregation approach to eliminate irrelevant data from the sensor network.

This approach works in three steps: (1) check similarity in sensor node level; (2) the sensor node data convert into groups using the *k*-mean algorithm; and (3) finally, check the human activity with SA score using Euclidean distance between cluster and centroid of data to decide whether to send it or not to the concerned sink.

The author [17] presents a cluster-based periodic sensor network (CPSN) data aggregation approach with aims to eliminate data redundancy and analyze the performance of data latency, accuracy, and energy consumption. This approach consists of two phases: local aggregation and cluster-based aggregation. In CH level, use three methods of distance functions, one-way ANOVA model, and set similarity function. The authors [18] have proposed a cluster-based data aggregation approach using the Comb-Needle model, which aims to minimize communication cost and energy consumption. The authors [19] have proposed a clustering approach in Underwater Sensor Network (UWSN) based on aggregation with Euclidean distance, aiming at data redundancy and analyzing network throughput and energy consumption. Author [11] proposed a periodic clustering approach for underwater in WSNs with the objective of efficient transmission and eliminate data redundancy. This approach is based on two tiers: one to eliminate redundancy in every period from sensing data if member nodes and the other for one-way ANOVA model using the *k*-mean algorithm with three statistical tests to eliminate data redundancy from the participant that make redundant data sets. The authors of [20] focuses on increasing network lifetime and reduce data transmission. For that, the two-phase protocol was proposed; in the first phase eliminate similarities between sensor nodes data, and in the second phase use distance function to find similarities between sets. This paper focused on decreasing data transmission that sensed by sensor nodes. For that, the authors were proposed a two-layer framework; the first layer divides nodes into clusters and the second layer is full sampling layer where data aggregation was fully performed that minimize the energy consumption of the network [21]. The authors proposed an efficient in-network approach for overcoming the whole transmitting data from member sensor nodes via CH to the base station; for that two-phase scheme was proposed, where in the first phase captured reading goes to an appropriate stratum and the range of stratum is decided; in the second phase two condition are checked, if the reading is minimum, then its compared with previous minimum reading where the smaller value will be next minimum value of stratum, and it should be minimum from new reading, the second condition is for maximum 3 value, the new value of reading compared with old maximum value and the greater value will be next maximum value for stratum [22].

RETRACTED

In [23], the authors have proposed a two-level approach for reducing temporal and spatial data redundancy from WSNs to enhance network lifetime and data reliability. The first level of the approach works on the end-node using the Kalman filter and the second level works on the base station using sink level algorithms. However, the energy consumption is high from existing schemes when compared and also no comparative analysis was done among all approaches. The authors have proposed a spatial correlation approach for the elimination of data redundancy from WSNs. The approach works on two levels: source and aggregator. The source level works based on similarity function and the aggregator works based on correlation technique. However, the loss of data is higher than other existing approaches when compared, and also no comparative analysis was done by the authors [24]. This study has proposed a data aggregation approach that uses less number of limited resources of sensor nodes to reduce data redundancy from WSNs. The approach works based on two levels: sensor node level and cluster head. The first level works based on Exponential Moving Average and threshold-based mechanism. The second level works based on an extended version of Euclidean distance. However, the proposed scheme shows high energy consumption when compared with other existing schemes [25]. The author has proposed a two-level data aggregation mechanism for WSNs to eliminate data redundancy to enhance network lifetime and save energy consumption. In the first level, cluster member nodes minimize data redundancy and also send error-free data to concerned CH. In the second level, *k*-mean algorithm is used for data aggregation. However, no comparative analysis was done [26].

RETRACTED

The authors work on reducing the redundant data and maintaining the integrity of data to send minimum data to the base station or final user and to achieve the above goals; the authors has used two phases method first local aggregation and the second is an aggregators level. Local aggregation used a link function to measure frequency and delete similarities. The aggregators level used the Jaccard similarity function for further aggregation [27]. The authors of the paper focused on increasing network lifetime and minimizing data redundancy for that proposed an Enhanced Clustering Hierarchy (ECP) approach. The objective of ECP is to overlap member nodes and use neighbors sleeping walking approach for minimizing data redundancy [28]. Redundant data use the network resources and decline the network performance by the congestion increasing. Due to the speedy growth of Internet data, various data redundancy methods have been proposed in recent years [29].

Many existing methods provided an appropriate solution to enhance the performance of the network by eliminating data redundancy from the network. It has been generally agreed that data redundancy elimination offers a huge advantage in practice. Usually, the advantage of eliminating the data redundancy is the enhanced network performance in terms of increasing throughput of the network and the decreasing end-to-end delay. However, the proposed techniques are not effective for eliminating redundant and irrelevant data from the network. For the above problem, we proposed a neighborhood-enabled scheme that solves related issues with resource-constrained network.

## 3. Proposed Neighborhood-Enabled Data Aggregation Approach for the IoTs

In this section, a detailed description of the proposed Neighborhood-Enabled and Cluster-Based Data Aggregation Scheme (NCDAS) is presented, which is designed specifically for the wireless sensor networks. The proposed approach bounds every CH module to refine data values, preferably through a neighborhood based aggregation mechanism, which are captured by the member devices. Actually, the proposed aggregation approach is based on the usual perception about member devices in IoTs that similarity index in data values captured by neighboring nodes is very high than other nodes. Therefore, the proposed scheme forces every CH module to compare data values of the nodes that are deployed in closed proximity in the IoTs. A detailed description of this mechanism is provided below.

RETRACTED

### 3.1. Network Model

Hierarchical wireless sensor networks are used where member nodes *C*_i_ are bounded to communicate via the respective CH module preferably those which are deployed in the coverage area with an approximate ratio of 1 : 20, as shown in Figure 1. Additionally, as the deployment process of WSNs is random, therefore, an imbalanced clustering approach is adopted where it is not necessary that every CH has equal number of member devices or nodes in the operational WSNs. Apart from it, Ad-Hoc On-Demand Distance Vector (AODV) protocol is used for the transmission of packets even if multiple nodes are eager to communicate simultaneously with the intended CH module. Likewise, User Data-Gram Protocol (UDP) is used as data communication protocol. Omnidirectional antenna model is used, whereas power consumption of packets transmission and receiving is 0.860 W and 0.5 W, respectively. Furthermore, packet size is 512 bytes and every member node is assumed to relay on it on-board battery.

### 3.2. Overview of the Proposed Scheme

Initially, every node has to capture data value after a defined time interval (i.e., 30 seconds in this case). As soon as data value is captured, it is transmitted to the intended destination devices, that is, nearest CH module in the proposed data aggregation and communication approach. Since every member node is assumed as a source device, then it is highly likely that CH module receives data values from multiple member nodes after the defined interval of time. Furthermore, CH module is bounded to transmit these data values to a centralized unit (i.e., server module or base station). However, before activation of the transmission activity, CH module needs to refine these values and checks it for possible noise and redundant data values. Generally, in IoTs, sensor nodes that are deployed in close proximity capture similar data values, and transmitting these redundant values is not only a wastage of resources but creates other problems, such as congestion and collision. Therefore, CH module is responsible for eliminating possible redundant data values and sends a refined version to the base station module. The proposed neighborhood-enabled data aggregation technique not only minimizes the ratio of redundant data values but at the same time avoids excessive matching of data values. For example, assume that CH module has received data values from nine member nodes as shown in Figure 2. In this figure, sensor node 1 has two closed neighbors, that is, sensor nodes 2 and 9. Generally, it is highly likely that data values captured by sensor node 1 are similar (approximately) to the data values captured by sensor nodes 2 and 9, which is due to the fact that these nodes are deployed in close proximity. However, data values captured by sensor node 6 are likely to be different from those of sensor node 1 or we can say similarity index between capture data values of sensor nodes 1 and 6 is very low or at minimum possible level in the IoTs. Therefore, matching captured data values of these two nodes, i.e., sensor nodes 1 and 6, is not only a wastage of time, as similarity index is very low, but seems not feasible as well as far as resource-limited nature of the IoTs is concerned. Thus, the proposed neighborhood-enabled data aggregation scheme not only refines data values captured by various member devices but at the same time avoids excessive matching or processing of irrelevant data in the IoTs.

RETRACTED

### 3.3. Neighborhood Discovery Phase

In this phase, a detailed description of the mechanism that is adopted in the proposed data aggregation approach to find neighboring devices or nodes in the operational IoTs is provided. For this purpose, every CH module is needed to broadcast a message with a hop count value equal to one in the payload. This message is received by those devices or nodes, which are deployed in close proximity or neighborhood to the concerned CH module in the IoTs. These nodes update or modify the received message parameters and rebroadcast them as soon as their backoff timer is expired. Backoff time is used to ensure a collision-free transmission of data values, preferably in scenarios where multiple devices or nodes are interested to communicate simultaneously. Backoff time is a random variable and is computed using the following equation.

(1) $$\begin{array}{c} \text{Backofftimer}=\text{rand}\left(20-1000\right). \end{array}$$

For example, if sensor nodes 4 and 5 are interested in sending an updated version of the received message, then it is highly likely that their packets will collide and retransmission will be required. However, if backoff timer is used, then it is highly likely that waiting time interval of these devices is different, which results in successful transmission of the updated packet in the IoTs. This mechanism is repeatedly applied by every CH module and sensor nodes until each and every device has collected information about neighboring devices in the IoTs. In addition to it, the proposed neighborhood-enabled scheme forces every sensor node to share its neighborhood information with the concerned CH module as well. This information is used by the respective CH module to decide which nodes data is needed to be matched to possible ratio of the redundant data values as shown in Figure 2. Furthermore, in order to understand the working mechanism (that is refinement of the captured data values) of the proposed neighborhood-enabled data aggregation scheme, a simplified workflow diagram is presented in Figure 3, where every step is depicted clearly. Every sensor node is assumed as a source device and is bounded to capture data values by interacting directly with the underlined phenomenon. Once the data is captured, then it is transmitted to the concerned CH module, preferably CH deployed in the coverage area of the transceiver module. As soon as the captured data values are received by the concerned CH module probably from different sources, then refinement or aggregation activity is initiated as shown in Figure 3. Data values of neighboring nodes are matched with each other to find redundant data values and eliminate them (if any exist). This mechanism is repeatedly applied to CH module after a defined time interval, and CH module sends a refined version, preferably with minimum possible redundant data values, to the concerned base station or server module. It is to be noted that the concerned CH module either sends the refined data directly to the respective base station or through multihop communication (if direct communication is not feasible). Apart from it, two data values particularly from different sources are assumed as similar if their difference or distance is less than a defined threshold value, that is, 0.1 in the proposed model, and it is computed using Euclidean distance measure as shown in the following equation, where *p* and *q* are two points.

(2) $$\begin{array}{c} d\left(p,q\right)=\sqrt{\left(q\;-\;p\right)2}. \end{array}$$

In the proposed neighborhood-enabled data aggregation approach, *k*-mean clustering is used to divide the deployed IoTs into clusters where it is not necessary that every cluster has similar member nodes (i.e., imbalanced clustering mechanism). In addition to the Euclidean distance measure, other distance measures are used to thoroughly examine their efficiency particularly from execution time, accuracy, and data refinement perspective. We have observed that support vector machine (SVM) is the best possible solution as far as efficiency of the proposed scheme is concerned in the IoTs.

RETRACTED

## 4. Proposed Neighborhood-Enabled Data Aggregation Algorithm

The proposed data aggregation algorithm has two phases, that is, (i) neighborhood discovery and (ii) refinement of data using *k*-mean clustering algorithm and SVM. It is to be noted that this algorithm is designed to be executed on the concerned cluster head module and is not feasible for the ordinary nodes due to their limited processing power capacities in the IoTs. After the deployment process of the IoTs, every node is bounded to become member of the nearest possible CH module in the IoTs, where ordinary nodes and CH modules are represented as N_*n* = {0, 1, 2, 3, N_n} and *k* = {k_1, *k*_2. . . k_n}, respectively. Every CH module is needed to broadcast a message with a hop count value equal to one in the payload. This message is received by those devices or nodes, which are deployed in closed proximity or neighborhood of the concerned CH module in the IoTs. These nodes update or modify the received message parameters and rebroadcast them as soon as their backoff timer is expired. Backoff time is used to ensure a collision-free transmission of data values preferably in scenarios where multiple devices or nodes are interested to communicate simultaneously. Backoff time is a random variable.

### 4.1. Neighborhood Identification Mechanism for Ordinary Nodes in the IoTs

In this section, a sophisticated mechanism to find neighboring devices or nodes of a particular member node is presented. As described in CH neighbor discovery section, every member node is forced to broadcast an updated version of message that is received from the nearest CH module in the IoTs. This message is not only received by the respective CH module, but it is also received by those nodes that are deployed in direct coverage area of the concerned node. For example, in Figure 2, message broadcasted by sensor node 8 is received by sensor nodes 7 and 9 as well in addition to the respective CH module. Therefore, these nodes assumed that sensor node 8 resides in close proximity and, thus, it is added to the neighboring node class. This mechanism is repeatedly applied by each and every sensor node in the operational IoTs. In order to further clarify, the proposed neighborhood-enabled aggregation approach allows CH module, as shown in Figure 2, to match data values of node 8 with the captured values of green-color nodes only. Similarly, for sensor node, data values of yellow nodes are matched against each other, whereas existing algorithms or techniques compare data values of one node against all possible member nodes in a given cluster. For cluster presented in Figure 2, CH is bounded to compare data values of sensor node one with captured data values of every other member node in this cluster (i.e., 2 to 9), which is time-consuming and costly.

### 4.2. Refinement of the Captured Data Using Euclidean Distance Measure

As described above, *k*-mean clustering is used to impose a hierarchical structure on the deployed nodes, preferably an imbalanced clustering approach. Additionally, *k*-mean clustering is used to refine the captured values that is received from multiple sources (i.e., sensor nodes in this case). To minimize the possible ratio of data redundancy, various distance measures (e.g., Euclidean, SVM, and *k*-mean clustering) have been utilized in the proposed neighborhood-enabled data aggregation mechanism. These methods are not only used to minimize duplicate data values but are equally utilized to improve lifetime of the underlined IoTs particularly with available resources. Sensor nodes are bounded to send data values to the concerned CH after a defined time interval, that is, sampling rate, in the IoTs. However, a tedious and time-consuming task for CH module is the identification of neighboring nodes, particularly whose data values are needed to be matched, that is necessary to avoid unnecessary comparison in the operational IoTs. For this purpose, Euclidean distance measure with a feasible threshold value is used to identify sensor nodes that reside in close proximity [30]. Thus, if distance between two member nodes is greater than the defined threshold value, then these nodes are assumed as nonneighbors and CH is forced to neglect these nodes while performing refinement of data values of the concerned member node or device in the IoTs (see Algorithm 1).

RETRACTED

### 4.3. Data Aggregation Using *k*-Mean and SVM Algorithms

As soon as the neighborhood discovery phase is completed, then every CH module has to eliminate (if possible) or reduce the possible ratio of the duplicate data values in the IoTs. The collected data is refined by the respective CH module through the neighborhood-enable aggregation approach as described above. However, it is highly likely that certain ratio of duplicate data values still exists even in the refined data set. Therefore, the proposed scheme has adopted two well-known algorithms, that is, *k* mean clustering and SVM classification, to further refine the underlined data sets by elimination duplicate data values. As both of these algorithms are computationally expensive, therefore only CH modules are bounded to apply these algorithms to the refined data sets to further improve accuracy and precision of the underlined decision support system. *k*-mean is a well-known clustering algorithm that has been proved as an effective way to find the redundant values in a given data set particularly those generated by sensor nodes in the IoTs. The key objective of the *k*-mean clustering algorithm is to create groups of clusters or data sets in such a way that data sets in the same cluster are very similar and data sets in different clusters are quite different. The key idea of *k*-means clustering is to organize *k* centroids in each cluster. The initial step is to take every point belonging to a specified data set and associate it with the closest centroid. The initial step is completed when no point is incomplete, and the initial grouping is finalized. After the first step, new k centroids are needed to be calculated for every cluster sequentially. When we get these *k* new centroids, a new binding has to be completed between the similar data set points and the closest new centroid. A loop has been made, and as a result of a loop, the *k* centroids change step by step their location until no further changes are done. After having recognized the final clusters that have redundant data sets, the CH removes redundancy from that cluster to decrease the amount of data transferred to BS. SVM is a machine learning algorithm that is used for regression or classification problems. However, SVM is typically used in classification challenges. In the context of our paper, we used SVM for classification purposes that divide nodes into two classes: redundant and nonredundant. The SVM classifications are primarily based on the following equation.

(3) $$\begin{array}{c} F\left(X\right)=T*C+N, \end{array}$$

where *N* is ID of sensor node, *C* is a constant value, and *T* is the threshold value.

(4) $$\begin{array}{c} H1=\left\{F\left(X\right)\leq 0\right\}\\ H2=\left\{F\left(X\right)>0\right\}. \end{array}$$

H1 and H2 are two hyperplanes, where one is greater than zero and another is less than or equal to zero. Actually, we have utilized equation (3) to separate the captured data into two classes, where 1 > 0 and 1 ≤ 0. Let us assume three support vectors (i.e., *S*_1_, *S*_2_, and *S*_3_). By integrating coordinates of the sensor nodes as described above, we get

(5) $$\begin{array}{c} S_{1}=\left(\begin{array}{c} X1\\ Y1 \end{array}\right),S_{2}=\left(\begin{array}{c} X2\\ Y2 \end{array}\right){\text{andS}}_{3}=\left(\begin{array}{c} X3\\ Y3 \end{array}\right). \end{array}$$

We assume bias value is 1.

(6) $$\begin{array}{c} S_{1}=\left(\begin{array}{c} X1\\ Y1\\ 1 \end{array}\right),S_{2}=\left(\begin{array}{c} X2\\ Y2\\ 1 \end{array}\right){\text{andS}}_{3}=\left(\begin{array}{c} X3\\ Y3\\ 1 \end{array}\right). \end{array}$$

Now, we take three parameters for the above vectors.

(7) $$\begin{array}{c} \alpha_{1}{\overset{⟶}{S}}_{1}{\overset{⟶}{S}}_{1}+\alpha_{2}{\overset{⟶}{S}}_{2}{\overset{⟶}{S}}_{1}+\alpha_{3}{\overset{⟶}{S}}_{3}{\overset{⟶}{S}}_{1}=1\\ \alpha_{1}{\overset{⟶}{S}}_{1}{\overset{⟶}{S}}_{2}+\alpha_{2}{\overset{⟶}{S}}_{2}{\overset{⟶}{S}}_{2}+\alpha_{3}{\overset{⟶}{S}}_{3}{\overset{⟶}{S}}_{2}=1\\ \alpha_{1}{\overset{⟶}{S}}_{1}{\overset{⟶}{S}}_{3}+\alpha_{2}{\overset{⟶}{S}}_{2}{\overset{⟶}{S}}_{3}+\alpha_{3}{\overset{⟶}{S}}_{3}{\overset{⟶}{S}}_{3}=1. \end{array}$$

So, we get the value of $\overset{⟶}{S}$_1,_$\overset{⟶}{S}$_2_, and $\overset{⟶}{S}$_3_.

(8) $$\begin{array}{c} {\overset{⟶}{S}}_{1}=\left(\begin{array}{c} X1\\ Y1\\ 1 \end{array}\right),{\overset{⟶}{S}}_{2}=\left(\begin{array}{c} X2\\ Y2\\ 1 \end{array}\right),{\overset{⟶}{S}}_{3}=\left(\begin{array}{c} X3\\ Y3\\ 1 \end{array}\right)\\ \alpha_{1}\left(\begin{array}{c} X1\\ Y1\\ 1 \end{array}\right)\left(\begin{array}{c} X1\\ Y1\\ 1 \end{array}\right)+\alpha_{2}\;\left(\begin{array}{c} X2\\ Y2\\ 1 \end{array}\right)\left(\begin{array}{c} X1\\ Y1\\ 1 \end{array}\right)+\alpha_{3}\;\left(\begin{array}{c} X3\\ Y3\\ 1 \end{array}\right)\left(\begin{array}{c} X1\\ Y1\\ 1 \end{array}\right)=1\\ \alpha_{1}\left(\begin{array}{c} X3\\ Y3\\ 1 \end{array}\right)\left(\begin{array}{c} X3\\ Y3\\ 1 \end{array}\right)+\alpha_{2}\;\left(\begin{array}{c} X2\\ Y2\\ 1 \end{array}\right)\left(\begin{array}{c} X2\\ Y2\\ 1 \end{array}\right)+\alpha_{3}\;\left(\begin{array}{c} X3\\ Y3\\ 1 \end{array}\right)\left(\begin{array}{c} X2\\ Y2\\ 1 \end{array}\right)=1\\ \alpha_{1}\left(\begin{array}{c} X3\\ Y3\\ 1 \end{array}\right)\left(\begin{array}{c} X3\\ Y3\\ 1 \end{array}\right)+\alpha_{2}\;\left(\begin{array}{c} X2\\ Y2\\ 1 \end{array}\right)\left(\begin{array}{c} X3\\ Y3\\ 1 \end{array}\right)+\alpha_{3}\;\left(\begin{array}{c} X3\\ Y3\\ 1 \end{array}\right)\left(\begin{array}{c} X3\\ Y3\\ 1 \end{array}\right)=1. \end{array}$$

After simplifying the above equation, the values of *α*_1_, *α*_2_, and *α*_3_ are computed for classes discriminates; the following equation is used.

(9) $$\begin{array}{c} \overset{⟶}{F}=\sum_{i=1}\mathrm{\alpha i}\overset{⟶}{S}. \end{array}$$

Put values in equation (4)

(10) $$\begin{array}{c} \alpha_{1}\left(\begin{array}{c} X1\\ Y1\\ 1 \end{array}\right)+\alpha_{2}\;\left(\begin{array}{c} X2\\ Y2\\ 1 \end{array}\right)+\alpha_{3}\;\left(\begin{array}{c} X3\\ Y3\\ 1 \end{array}\right)=\left(\begin{array}{c} \alpha 1X1+\;\alpha 2X2+\;\alpha 3X3\\ \alpha 1Y1+\;\alpha 2Y2+\alpha 3Y3\\ \alpha 1+\alpha 2+\;\alpha 3 \end{array}\right). \end{array}$$

in $\left(\begin{array}{c} \alpha 1X1+\;\alpha 2X2+\;\alpha 3X3\\ \alpha 1Y1+\;\alpha 2Y2+\alpha 3Y3\\ \alpha 1+\alpha 2+\;\alpha 3 \end{array}\right)$.

*α*_1_ + *α*_2_ + *α*_3_ is the threshold value that is used for separation of classes in equation (3).

RETRACTED

## 5. Experimental Results

In order to evaluate and verify effectiveness of the proposed NCDAS, extensive simulations in terms of various performance metrics have been performed, such as packet delivery ratio, network lifetime, energy consumption, throughput, and end-to-end delay. For comparison, we have compared the performance of the proposed data aggregation approached against the latest field proven approaches, such as [16, 17, 31, 32]. These algorithms were implemented in network simulator 2 (NS-2) using similar topological infrastructures. Apart from this, these approaches were thoroughly checked for varying sensor nodes, threshold values, and readings. Various parameter used in the simulation setup are presented in Table 1.

### 5.1. Data Aggregation at CH

Cluster head is assumed as one of the core components of the heterogeneous WSNs as majority of the processing is carried out at this level. Therefore, it is mandatory to evaluate the performance of the proposed data aggregation scheme at this level. In the proposed data aggregation approach, CH is not only responsible for refining the capture data values of its member devices but at the same acting as destination devices for member devices as well. Simulation results show that the performance of the proposed data aggregation scheme is far more better than the existing state-of-the-art approaches, as depicted in Figure 4. From Figure 4, we have observed that *k*-mean and SVM with embedded neighborhood-enabled (proposed) approach aggregates or refine the captured data values up to 66.23% and 45.28%, respectively, whereas the aggregation ratio of IDK, SVM, Euclidean distance, cosine distance, and NCDAS approches are 69.56%, 55.56%, 56.24%, 57.56%, and 70.23%, respectively. However, 100% data is sent to the BS if no aggregation activity is performed. In terms of data redundancy or duplication, the proposed neighborhood-enabled approach eliminates 98.4% of the duplicate data values.

### 5.2. Energy Efficiency at CH

Energy efficiency is assumed as an essential component to evaluate the performance of the newly developed algorithm, specifically those that are designed for the wireless sensor networks. It is due to the fact that member devices in these networks solely rely on the on-board batteries; thus, prolonged lifetime of both individual device and whole network is highly appreciated by the research community. For this purpose, we have evaluated energy consumption of the proposed and existing approaches at the CH level, which is bounded by the proposed scheme to refine the captured data values of its member devices or sensor before sending it to the gateway module. Simulation results clearly depict that the average energy consumption of the proposed scheme is far better than the existing state-of-the-art schemes particularly at CH level in the IoTs. Furthermore, we have observed that the NCDAS, specifically when not embedded with the *k*-means and SVM algorithms, consumes 6.55 J, with *k*-mean and SVM 8.1 8.54 J of the on-board battery, respectively, at CH, whereas IDK, SVM, cosine distance, and Euclidean distance are 8.6789 J, 9.1 J, 8.92 J, and 8.76 J, respectively, as shown in Figure 5. Likewise, when the proposed scheme is integrated with the *k*-mean to form a hybrid refinement mechanism, then the simulation results show that its performance is according to the expectations, that is, better than existing state-of-the art approaches. The proposed approach when merged with the *k*-mean has less energy consumption from a hybrid of proposed scheme and SVM (i.e., 5.15%), from IDK is 6.77%, from SVM is 10.98%, from Euclidean distance is 7.53%, and from cosine distance is 9.19%.

RETRACTED

### 5.3. End-to-End Delay

The end-to-end delay of the NCDAS is 1.532 ms, which is less than from existing schemes and proposed hybrid schemes. The proposed scheme with *k*-mean has an end-to-end delay of 2.92 ms and the proposed with SVM is 1.87 ms, whereas end-to-end delay of IDK, SVM, Euclidean distance, and cosine distance are 3.41 ms, 2.11 ms, 2.96 ms, and 1.96 ms, respectively. The proposed scheme when integrated with the SVM approach is 35% than proposed with *k*-mean, 45% from IDK, 37% from Euclidean, 6% from SVM, and 12% from cosine are lesser when compared with these approaches (Figure 6).

### 5.4. Average Packet Delivery Ratio (APDR)

APDR is considered as an important evaluation metric to judge the performance of the newly developed approach using well-known topological infrastructures. To evaluate the performance of the proposed data aggregation approach, specifically in terms of APDR, the proposed scheme along with existing approaches is implemented in realistic environment of IoTs. During the simulations, we have observed that the APDR of the NCDAS is better than the existing state-of-the art schemes as shown in Figure 7. APDR of the proposed scheme is integrated with *k*-mean is 87.21% and with SVM is 90.21%, where IDK is 68.58%, SVM is 87.11%, Euclidean distance is 86.24%, and cosine distance is 65.15%. The ratio of the NCDAS is 93.22%, which is good from other schemes. The PDR of proposed scheme with SVM is 3.44% from proposed with *k*-mean, 31.53% from IDK, 3.5% from SVM, 4.60% from Euclidean distance, and 38.46% from cosine distance are higher when compared with these schemes.

### 5.5. Throughput

The throughput of the sensor network is defined as the ratio of packets that are delivered successfully to the intended destination device (i.e., the base station in this case). Additionally, it is to be noted that we have assumed that IoTs become inactive as soon as the very first node consumes its on-board battery completely. Throughput analysis of the NCDAS and existing schemes is shown in Figure 8, which depicts that the proposed scheme has a relatively higher throughput than the existing state-of-the-art schemes. Likewise, the proposed scheme performance, specifically in terms of throughput, is improved further if it is integrated with the *k*-mean than the hybrid of the proposed SVM, proposed IDK, proposed SVM, proposed Euclidean, and proposed cosine, respectively. Apart from it, we have observed that a hybrid of the proposed *k*-mean performs better in terms of packet loss ratio, which is 1.54%. Similarly, when the proposed scheme is integrated with SVM, then packet loss ratio is 12.84%, which is better than that IDK, SVM, and Euclidean i.e., 19.12%, 5.54%, and 52.54%, respectively.

RETRACTED

### 5.6. Network Lifetime

Lifetime is one of the critical and vital evaluation metrics that is used by the research community to examine the performance of the newly developed scheme for the IoTs and other resource-constrained networks. Network's lifetime of the proposed neighborhood-enabled data aggregation and existing state-of-the-art schemes is presented in Figure 9. During the simulation setup of the proposed data aggregation approach, we have observed that the NCDAS approach and the proposed integrated with SVM leads to the minimum possible set of dead nodes (i.e., 16 and 23 in this case). Similarly, the proposed scheme is when integrated with the *k*-mean; then death ratio of member devices is 35. Likewise, for IDK, SVM, and cosine, the ratio of dead nodes is 33, 51, and 42, respectively. Additionally, the proposed with SVM is an ideal solution, which is depicted in Figure 9. Moreover, the proposed scheme when combined with the *k*-mean, its dead-to-alive node ratio is 34.28%, from IDK is 30.30%, from SVM is 53.06%, from Euclidean distance is 45.38%, and from cosine is 39.47% when these approaches are compared.

### 5.7. Normalized Routing Overhead

In Figure 10, the normalized overhead of proposed neighborhood-enabled data aggregation and existing schemes is presented. It shows that the NCDAS has less normalized overhead than the existing schemes. The normalized overhead of proposed when integrated with *k*-mean is 1.19 and with SVM is 1.015, where with IDK is 1.45, SVM 1.35, Euclidean distance 1.16, and cosine distance is 1.56. The NCDAS overhead is 1.001, which is less from other schemes when compared with these schemes.

## 6. Comprehensive Comparison of the Proposed and Existing State-of-the-Art Schemes

The aim of this comprehensive study is to compare the proposed scheme with existing ones, to find which scheme is best among all. Here, we compare the NCDAS and proposed with SVM and *k*-mean with four existing schemes. The performance metrics values of all schemes are presented in Table 2. Based on the results of Figure 4, the proposed with SVM is giving the best result in data aggregation, where all evaluation parameters suggest that the proposed with SVM aggregate data accurately among all. In Figures 5 and 8, it is presented that the NCDAS and the proposed with *k*-mean in terms of energy consumption is the lowest, and in terms of throughput of the network, it is higher among all schemes. Based on the result of Figures 10 and 6, it shows that the NCDAS and the proposed with SVM in terms of normalized routing overhead and end-to-end delay is the lowest among all schemes. In Figure 7, the packet delivery ratio is shown in all schemes such that the NCDAS and the proposed with SVM has a good packet delivery ratio among all. The proposed with SVM in terms of network life is good based on results shown in Figure 9; the number of dead nodes during simulation time is smaller among all when compared. The performance metric results of all schemes when compared to that of the proposed scheme have the best results among all aspects.

RETRACTED

## 7. Complexity Analysis of the Proposed and Existing State-of-the-Art Schemes

In this section, we discuss all scheme time complexity, which is shown in Table 3. We consider the time complexity of all schemes, which are used in the data aggregation phase and the reason is that the previous papers only consider the data aggregation algorithm time complexity. The Euclidean and cosine distance has (Θ(n2)) time complexity and IDK have Θ(n2)*∗*Θ(n) [16, 17, 32], where the SVM [31] time complexity is Θ(n) *∗*Θ(3n); the proposed with *k*-mean and proposed with SVM have Θ(n) *∗*Θ(n) and Θ(n)*∗*Θ(n) *∗*Θ(3n) time complexity; here in proposed with SVM we did not consider the training timing complexity, only considering the classification time complexity of the work. The NCDAS has Θ(n); based on the above results, the proposed has the best time complexity among all when compared.

## 8. Further Discussion

In this section, we give further explanations of our proposed schemes. In the experimental section, we saw the comparison of existing and proposed schemes while applying. The performance of all schemes is evaluated based on performance metrics. From data aggregation and redundancy point of view, the proposed scheme with SVM gives the best result among the other schemes and actual data reduce to 45.28%. The proposed with SVM more reduces data from proposed with *k*-mean 31.63%, from IDK is 34.90%, from SVM is 18.50%, from a Euclidean distance is 19.48%, from cosine distance is 21.33%, and from NCDAS is 35.536% when these schemes are compared.

RETRACTED

In terms of energy consumption, the NCDAS and the proposed with *k*-mean consume less energy at CH among other schemes; the proposed scheme saves more energy compared to other schemes. The NCDAS saves energy, that is, 30.38% from proposed with SVM, from the proposed with *k*-mean 23.66%, from IDK 32.48%, from SVM 61.06%, from Euclidean distance and cosine distance are 36.18% and 33.74% when compared with these schemes in terms of energy consumption at CH. From the end-to-end delay point of view, we see that the NCDAS and the proposed with SVM scheme give a good result in terms of the end-to-end delay among others when compared with Euclidean distance, cosine distance, SVM, IDK, and proposed with *k*-mean schemes. The Euclidean distance and IDK give the highest end-to-end delay from other schemes; the Euclidean from proposed with SVM is 37% where IDK is 45%. We see that SVM and cosine distance also give minimum end-to-end delay from IDK, Euclidean distance, and proposed with *k*-mean. From the packet delivery ratio point of view, the proposed with SVM and the NCDAS gives the highest delivery ratio among other schemes when these schemes are compared. The PDR of proposed with *k*-mean and SVM are higher than Euclidean distance, cosine distance, and IDK. The lowest delivery ratio is of cosine distance, which is 65%. From the throughput point of view, the proposed with *k*-mean has the highest throughput among other schemes. We see that IDK also has good throughput from other schemes in terms of lowest throughput is of cosine distance, which is 42.1 Mbps. The result of SVM, particularly when combined with the proposed scheme, are better than Euclidean distance and SVM as shown in the results section. From the network lifetime point of view, the NCDAS and the proposed with SVM have a good network lifetime among other schemes. We see that the cosine distance and SVM have not a good network lifetime when compared with other schemes. The proposed with SVM is considered the best scheme among all in terms of data aggregation, energy consumption, delay, delivery ratio, and network lifetime. Based on the above results, our proposed scheme is best for a large and small network. The user can use this scheme in his own interest; in this paper, we did not consider the integrity of data; in general, data are secured and without any loss are sent to the base station.

Although the proposed data aggregation scheme has resolved the challenging issue of the redundant data in the data which is captured by the various sensor nodes deployed in closed proximity of the phenomena, however, a common issue with the proposed approach and other data aggregation approaches is that these approaches have compromised on data loss of the smallest possible portion of the underlined data. Although the proposed approach is very effective in reducing the ratio of duplicate data values, a significant portion of data is lost. Finally, in the proposed data aggregation approach, every sensor node along with cluster head module is bounded to compute or find its neighborhood information, which consumes a significant portion of the available power. Moreover, this process is time-consuming specifically in situations if deployment density of the underlined sensor nodes is very densed.

RETRACTED

## 9. Conclusion

In this paper, we have proposed a neighborhood-enabled and machine learning-enabled data aggregation scheme for the resource-constrained network. In our proposed approach first, we find neighbors in the cluster and then use data aggregation and redundancy check at CH level, where data comes from member sensor nodes that sense the physical environment. When neighbor nodes are found, then data redundancy check only with neighbor nodes and then *k*-mean and SVM data aggregation algorithms are applied on remaining data, which further clean data. After using data aggregation, the refined data are sent to the base station. We see that our approach extends network lifetime, increases throughput and packet delivery ratio, and decreases energy consumption and the end-to-end delay. In the future, this scheme will be used on real data set for more validation and evaluate this scheme with real-time data aggregation schemes.

## Figures and Tables

**Figure 1:** Proposed network topology for data aggregation.

**Figure 2:** Aggregation at CH.

**Figure 3:** Proposed scheme for data redundancy elimination.

**Figure 4:** Data aggregation at CH of the proposed versus existing state-of-the-art schemes.

**Figure 5:** Average energy consumption at CH of the proposed versus existing state-of-the-art schemes.

**Figure 6:** End-to-end delay of the proposed versus existing state-of-the-art schemes.

**Figure 7:** Packet delivery ratio of the proposed versus existing state-of-the-art schemes.

**Figure 8:** Throughput of the proposed versus existing state-of-the-art schemes.

**Figure 9:** Number of alive nodes in proposed scheme versus existing state-of-the-art schemes.

**Figure 10:** Normalized overhead of the proposed versus existing state-of-the-art schemes.

**Algorithm 1:** NCDAS Algorithm.

**Table 1:** Simulation parameters.

Routing protocol	AODV
Number of nodes	100
Network size	1000 × 1000 m
MAC protocol	IEEE 802.11
Antenna model	Omnidirectional antenna
Initial energy	10.0 J
Transmission power	0.860 W
Receiving power	0.5 W
Packet size	512 bytes

RETRACTED

**Table 2:** A detailed comparative analysis of the proposed and existing state-of-the-art schemes.

Schemes	Data aggregation	Energy consumption (J)	End-to-end delay (ms)	Normalized overhead	PDR (%)	Throughput (Mbps)	Dead nodes
NCDAS	70.23%	6.55	1.532	1.001	93.22	66.26	16
Proposed with SVM	45.28%	8.54	1.87	1.015	90.21	63.22	23
Proposed with *k*-mean	66.23%	8.1	2.92	1.19	87.21	64.22	35
IDK	69.56%	8.678	3.41	1.45	68.58	63.84	33
SVM	55.56%	9.1	2.11	1.35	87.11	53.91	51
Euclidean distance	56.24%	8.92	2.96	1.16	86.24	60.84	42
Cosine distance	57.6%	8.76	1.96	1.56	65.15	42.01	38

**Table 3:** Complexity analysis of the proposed and existing schemes.

Schemes	Time complexity
NCDAS	Ө(n)
Proposed with SVM	Θ(n) *∗*Θ(n) *∗*Θ(3n)
Proposed with *k*-mean	Θ(n) *∗*Θ(n)
IDK	Ө(n2)*∗*Ө(n)
SVM	Ө(n)*∗*Ө(3n)
Cosine distance	Ө(n2)
Euclidean distance	Ө(n2)

## Data Availability

The data sets used and analyzed during the current study are available from the corresponding author upon reasonable request.
